The article "Therapeutic Investigation of Standardized Aqueous Methanolic Extract of Bitter Melon (Momordica charantia L.) for Its Potential against Polycystic Ovarian Syndrome in Experimental Animals' Model: In Vitro and In Vivo Studies" was published in 2022. Journal: Evid Based Complement Alternat Med.

# Therapeutic Investigation of Standardized Aqueous Methanolic Extract of Bitter Melon (*Momordica charantia* L.) for Its Potential against Polycystic Ovarian Syndrome in Experimental Animals' Model: *In Vitro* and *In Vivo* Studies

**DOI:** 10.1155/2022/5143653

**Published:** 2022-09-29

**Authors:** Liaqat Hussain, Noor Aamir, Musaddique Hussain, Muhammad Asif, Zunera Chauhdary, Faiza Manzoor, Rida Siddique, Muhammad Riaz

**Affiliations:** ^1^Department of Pharmacology, Faculty of Pharmaceutical Sciences, Government College University Faisalabad, Faisalabad, Pakistan; ^2^Department of Pharmacology, Faculty of Pharmacy, Islamia University Bahawalpur, Bahawalpur, Pakistan; ^3^Department of Nutritional Sciences, Faculty of Medical Sciences, Government College University, Faisalabad, Pakistan

## Abstract

Polycystic ovarian syndrome (PCOS) is an heterogenous, endocrine, metabolic, and multidisciplinary disorder of reproductive-aged females that aggravates insulin resistance, hyperandrogenism, obesity, menstrual irregularities, and infertility. Bitter melon is consumed as vegetable in various parts of the world. The purpose of this study was to provide the rationale for the folkloric uses of bitter melon *(Momordica charantia* L.) in reproductive abnormalities. HPLC analysis of standardized aqueous methanolic extract of bitter melon revealed the presence of various phytochemicals such as quercetin, gallic acid, benzoic acid, chlorogenic acid, syringic acid, *p*-coumaric acid, ferulic acid, and cinnamic acid. Twenty-five Swiss albino adult female rats (120–130 g) were acquired and divided into two groups (5 + 20). Letrozole (1 mg/kg *p.o*.) was used for four weeks to induce PCOS in twenty rats. Disease induction was confirmed by vaginal smear cytology analysis under the microscope. Animals were further divided into four groups, with one group as PCOS group, and the remaining three are treated with standardized extract of bitter melon (500 mg/kg *p.o.*), bitter melon plus metformin (500 mg/kg *p.o.*), and metformin alone for the period of next four weeks. After four weeks, the rats were euthanized at diestrus stage. Ovaries of the experimental animals were removed and fixed in 10% buffered formalin, and blood samples were obtained from direct cardiac puncture and stored. Ovaries histopathological analysis showed cystic follicles (9–10) in PCOS group, while, in all the treatment groups, we found developing and mature follicles. Similarly, hormone analysis showed significant (*p* < 0.001) reduction of LH surge, insulin, and testosterone levels and improvement in FSH levels. Lipid profile and antioxidant enzymes status were also significantly (*p* < 0.001) improved. In conclusion, the study validates the bitter melon potential as an insulin sensitizer and ovulation enhancer and authenticates its potential in PCOS management.

## 1. Introduction

Polycystic ovarian syndrome, commonly known as PCOS, affects the females during their early to late reproductive age and is considered as a disorder that causes infertility, anovulation, and hyperandrogenism [1]. PCOS mainly affects at least 5–10% of the females and is mostly distinguished by various signs and symptoms such as hormonal dysregulation, irregular menstrual cycles, and dysfunction of follicular maturation, and in some cases also miscarriages [2]. If we access the prevalence on the basis of broader Rotterdam Criteria, the ratio is as high as 15% [3]. Because of the dysregulation of follicular stimulating hormone (FSH) and luteinizing hormone (LH), females might suffer from conditions such as hirsutism and acne [4].

Due to this endocrine abnormality, affected individuals have to face multiple physical, psychological, social, and economic issues [5]. This endocrine abnormality might be due to weight gain, insulin resistance, or androgen-secreting neoplasms. Hyperandrogenism and hyperinsulinemia have been found to coexist in PCOS. Insulin interacts synergistically with LH, resulting in hyperthecosis and decreased hepatic production of sex hormone binding globulin (ShBG), which enhances anovulatory processes [6]. The revised definition of PCOS is based on clinical and biochemical parameters and ovarian morphology. It is established that women who have regular cycles and hyperandrogenism might be fulfilling the criteria of this definition. PCOS is diagnosed if two of the following parameters are present:

- polycystic ovaries;
- oligo or anovulation;
- clinical or biochemical evidence of hyperandrogenism [3].

PCOS management is quite irrigating, and there are interindividual differences and mostly depends upon symptomatology [7]. Lifestyle modification is one of the recommended strategies in obese individuals including mild-to-moderate exercise, weight management, and caloric intake reduction, reducing stress and decreasing caffeinated beverages [8, 9]. The treatment option mostly adopted is metformin, pioglitazone, estrogen, and progesterone combination (oral contraceptives; OCPs), GnRH agonist, myo-inositol, and various evolution enhancers such as letrozole and clomiphene citrate [10–12]. But none of these agents are free of side effects; hormonal therapies and pioglitazone cause wight gain, cardiovascular abnormalities and metformin cause lactic acidosis, and OCPs cause lower abdominal pain and dysmenorrhea [13].

In recent times, we have seen health care systems that recognized the importance of food-based, alternative, and complimentary medicines. This incline is might be due to better awareness of toxicity profile of all the above allopathic regimens or due to higher cost [14, 15]. Phytochemicals present in herbal remedies and medicinal plant are source of therapeutic effectiveness against the ailment such as PCOS [16, 17]. It is really a remarkable thing that herbal therapy for PCOS always proved their effectiveness in improving insulin sensitivity, enhancing ovulation, and reducing hyperandrogenism without toxicity that is discussed above. Due to these reasons, individuals are more satisfied with herbal remedies. Various herbal and alternative interventions are used for PCOS such as *Aloe vera*, cinnamon, *Glycyrrhiza glabra*, *Mentha spicata*, *Panax ginseng*, *Fagonia indica*, flaxseed, N-acetyl cysteine, and inositol [9].

One common plant (*Momordica charantia* L.) (family: Cucurbitaceae), commonly known as bitter melon, is an indigenous medicinal plant and vegetable that can be found in most parts of the world [18]. It has gained an enormous fame for its use in diabetes, due to its biological activity to maintain the glycemic levels of diabetic patients [19]. In addition to diabetes, it has pharmacological activity against cancer [20], cough, colic and stomach pain [21], constipation, asthma, leprosy [22], gout, helminthiases, malaria fever, wound healing [23], ulcers [20], antimicrobial, and inflammation [22]. Bitter melon has been used traditionally for diabetes, various metabolic disorders, and also menstrual abnormalities for many years. Thus, this present study is aimed to provide rationale for the folkloric uses of bitter melon especially in metabolic syndrome like PCOS. Therefore, in this study, we explored the pharmacological potential of standardized aqueous methanolic extract of bitter melon by using female adult Swiss albino rats after inducing PCOS with letrozole.

## 2. Material and Methods

### 2.1. Collection and Authentication of Plant

Fresh bitter melon fruit, also known as *Momordica charantia* L., was collected from vicinity of Faisalabad, Pakistan. The fruit was washed properly and identified from taxonomist Dr. Qasim Ali, Assistant professor, Department of Botany, Government College University, Faisalabad. A voucher number: 277-bot-21 was submitted in concerned herbarium for future reference.

### 2.2. Preparation of Extract

Fresh bitter melon fruit was treated with tap water to remove the excess dirt, pat-dried in folds of filter paper, and cut into equal segments with the seeds inside the fruit. The fruit was air-dried until all the moisture content was removed and converted into powder. One kg of each plant material was soaked in 30% water and 70% methanol at 1 : 5 proportions and placed for 7 days for proper soaking and maceration. The soaked mixture was shaken every day at different time intervals. A muslin cloth was used to remove the large particles from the mixture, and then, the mixture underwent filtration using Whatman No. 1 filter paper [9]. The filtrate accumulated after resoaking the material in 70% methanol twice for above mentioned time period was set up on a rotary evaporator (Scilogex RE100-pro 5 L) to remove the excess solvent to obtain a thick semisolid mass. This was stored in airtight containers for future usage in freezer at −20°C.

### 2.3. Extract *In Vitro* Analysis

#### 2.3.1. Extract Characterization by HPLC Analysis

HPLC method was developed for the contemporaneous quantitative findings of quercetin, gallic acid, benzoic acid, chlorogenic acid, syringic acid, *p*-coumaric acid, ferulic acid, and cinnamic acid in fraction of bitter melon (*Momordica charantia* L.). In order to obtain good separation with HPLC, acetic acid was used in the ratio of around 94 : 6 v/v pH = 2.27, and acetonitrile 100% was regarded as the mobile phase. Densitometric identification was performed at 280 nm in absorption mode. Linear calibration curve with a scale of around the range of 100–400 mg/spot was used for all the above mentioned phytoconstituents. The suitable and improved method was intentionally used for the evaluation of three major phenolics in the case of bitter melon extract. The suggested procedure in this case was relatively easy, explicit, and meticulous, as well as more accurate and correct [24].

#### 2.3.2. Total Phenolic Content (TFC)

The technique of Singleton and Rossi with modifications was used for the determination of the total phenolic content of bitter melon extract. The established protocol followed the one used in our previous study [9, 25].

#### 2.3.3. Total Flavonoid Content (TPC)

Total flavonoid contents of bitter melon extract have been evaluated by the method of Wang and collogues [26]. Two mL of distilled water was mixed with 0.5 mg of extract and 0.15 ml of sodium nitrate (5%) solution. Incubation was done for six minutes. Aluminum chloride (10% of 0.15 mL) and 4% sodium hydroxide admixed with solution were used alternatively after this 6-minute incubation again. Methanol (95%) was added to make volume of reaction mixture up to 5 mL. After incubation for 15 minutes, absorbance was taken at 510 nm. Total flavonoid contents (TFC) of plant extract were represented as catechin equivalents [27].

### 2.4. Experimental Animals' Housing

Adult female Swiss albino rats (*N* = 25) weighing 120–130 g were gained from the animal house of Government College University, Faisalabad. A pathogen-free barrier facility along with a controlled environment was provided to the animals. The animals were provided standard 12 h light/dark cycle with water *ad libitum* (temperature: 25 ± 2°C, relative humidity: 45 ± 5%), and standard diet was provided. All the *in vivo* experiments were conducted according to guidelines of animal use for experimental purpose as recommended by the European Union on Animal Care. The pre-study approval was obtained from the Ethical Review Committee (ERC) of Government College University Faisalabad and was further permitted by Advance Studies and Research Board (ASRB).

### 2.5. Disease Induction

Before the start of the experiment, the animals were acclimatized for a week and daily monitoring through vaginal smears observed under the microscope to assess the estrous cycle stage. In diestrus stage, PCOS disease induction was initiated. Any experimental animal that was observed to have a missed or irregular estrous cycle was excluded from the study. Initially, the animals were divided into two groups: Normal Control group (N.C, *n* = 5) and Disease Induced Group (PCOS group, *n* = 20). N.C was administered 0.5% carboxyl methylcellulose solution (CMC) 10 mL/kg/day), and PCOS group was administered letrozole (1 mg/kg/day *p.o*.) dissolved in CMC and continued for around 4 weeks [28]. During the disease induction period, the estrous cycle was monitored daily by vaginal smear cytology (presence of cornified cells, leukocytes, and epithelial cells in relative proportion under light microscope), and weight variations was also recorded. The study exclusion criteria were based on the cyclic regulation of estrous cycle, no weight gain, and the normalization biochemical parameters.

### 2.6. Experimental Design

After disease induction, PCOS induced group was randomly divided into four more groups (5 animals/group), 2^nd^ group as PCOS (positive control), 3^rd^ group on bitter melon (*Momordica charantia* L.), 4^th^ group on bitter melon plus metformin, and 5^th^ group on metformin alone. The detailed experimental design is given in Table 1. Doses were administered daily, and vaginal smear was examined by microscope [29].

#### 2.6.1. Sample Collection Procedure

At the end of every week, animals were weighed. At the end of four weeks, after 24 hours of the last dose, all animals were euthanized, and blood samples were collected by cardiac puncture. The serum was separated by centrifuge machine, frozen at −20°C for hormonal and biochemical analysis. Both ovaries were removed for histopathological analysis. Liver was removed and preserved in 10% buffer formalin to check the antioxidant status. [29–32].

#### 2.6.2. Estrous Cycle Monitoring

Female albino rats estrous cycle contains four stages: proestrus, estrus, metestrus, and diestrus. Proestrus stage consists of oval, well-formed, nucleated epithelial cells. Estrus stage dominated with cornified squamous nucleated cells. Metestrus stage comprises a small number of leukocytes and nucleated epithelial cells along with cornified epithelial cells, while the diestrus phase mostly contains leucocytes and mucus. The female rats were individually handled, and a cotton swab soaked in normal saline was inserted through vaginal route. A thin smear was taken on glass slides and stained with methylene blue for better results [33]. The slides were observed under the microscope to determine the stage of the estrous cycle of each individual rat.

#### 2.6.3. Histopathological Observation of Ovaries

As discussed in the upper section, ovaries of each rat were isolated, cleaned, and fixed in 10% buffer formalin solution. The ovaries were washed to remove formalin, and dehydration was done with isopropyl alcohol at variable strength (70%, 80%, and 90%) for a time of 12 h for each strength. Again, we performed dehydration with absolute alcohol for the same duration [34]. After fixation, paraffin blocks of 5 *µ*m thickness were designed, and microtome was used to cut down slices according to blocks. Slides were prepared, and staining was done with eosin and hematoxylin and analyzed under microscope (Accu-Scope 3000).

#### 2.6.4. Serum Hormone Analysis

The blood samples were centrifuged at 2500 rpm for 10 minutes to collect serum, so that it can be utilized for hormone analysis tests, for example, insulin, testosterone, progesterone, FSH, and LH. Enzyme-linked immunosorbent assay (ELISA) kit (MLBio, Shanghai, China) method was adopted for analysis of serum LH and insulin. For each assay, intra- and interassay coefficients of variation were  <10% and  <15%, respectively. Optical density values were read at 450 nm using a microplate reader. Estimation of serum FSH, progesterone, and testosterone levels were determined by radioimmunoassay (RIA; Beckman Coulter Inc. USA). IR was appraised with the homeostasis model assessment of insulin resistance (HOMA-IR) method [35].

#### 2.6.5. Lipid Profile

Lipid profile assessment was done, and various lipid markers were determined, that is, total serum cholesterol, triglycerides, HDL, and LDL. Automated chemistry analyzer (Microlab-300) was used to perform lipid profile estimation.

### 2.7. Antioxidant Activity Assessment

#### 2.7.1. Determination of Enzymatic Activity

In PCOS, the levels of antioxidant enzymes, for example, catalase (CAT) and superoxide dismutase (SOD), are mostly altered [36]. Thus, we appraised their level in the current study. The liver tissues were utilized, and liver homogenates were prepared by using 0.1 M phosphate buffer saline (pH 7.4). The mixture was centrifuged for 30 min at 800 rpm at 4°C to obtain the supernatant. The antioxidant enzymes concentration was obtained by using this supernatant solution [37].

#### 2.7.2. DPPH Radical Scavenging Assay

DPPH radical scavenging assay was performed to assess the antioxidant potential of the extract. This was done according to established protocols, already published, and we also used the same protocols in our previous studies [9, 32, 37, 38].

### 2.8. Statistical Analysis

The data were presented as mean ± SEM, and the results of different groups were compared by analysis of variance (ANOVA) using GraphPad Prism 8.0.2, followed by Tukey's multiple comparisons test. The results were considered statistically significant if the *p* value was less than 0.05.

## 3. Results

### 3.1. Extract *In Vitro* Analysis

#### 3.1.1. Phytochemical Quantitative Analysis by HPLC Analysis

HPLC (model SPD-10AV with a UV-visible detector made by Shimadzu, Japan) was used to analyze the presence of phytoconstituents present in the aqueous methanolic extract of bitter melon (*Momordica charantia* L.). The extract contains only flavonoids such as quercetin and phenolic compounds such as gallic acid, benzoic acid, chlorogenic acid, syringic acid, *p*-coumaric acid, ferulic acid, and cinnamic acid. The HPLC chromatogram is displaying various minor and major peaks (Figure 1). The phytoconstituents names, as identified by the absorbance rates and retention time and given in parts per million (PPM), all are mentioned in Table 2. The structures of few phytochemicals are drawn in Figure 2.

#### 3.1.2. Total Phenolic Content (TFC) and Total Flavonoid Content (TPC)

The aqueous methanolic extract of bitter melon (*Momordica charantia* L.) contains a rich proportion of TFC, and it was calculated to be 343.87 ± 3.89 mg GAE/g, expressed as gallic acid equivalent, while bitter melon extract also contains flavonoids, and the amount calculated was 404.60 ± 4.99 mg CE/g, expressed as catechin equivalent.

### 3.2. *In Vivo* Studies

#### 3.2.1. Monitoring of Estrous Cycle

The estrous cycle monitoring was done for Normal Control (NC) and PCOS induced group to confirm the induction of the disease. The vaginal smears were observed under microscope, and the stage of the estrous cycle was confirmed. Mainly, the stages were called 1, 2, 3, and 4 (proestrus, estrus, metestrus, and diestrus, respectively) as shown in Figure 3. The observation was carried out for a period of 28 days. The PCOS induced group showed irregular stages, which clearly indicates the induction of PCOS, whereas the normal control group was observed to have a normal regular cycle.

#### 3.2.2. Effect of Bitter Melon Extract on Histopathology of Female Rat Ovaries

All the female rats were euthanized, and the ovaries were removed as mentioned earlier in the Materials and Methods. The tissues slides of each group were prepared and observed under different resolutions of a microscope to determine the histopathological changes that took place under the influence of plant extract on the PCOS induced female rats. When the Normal Control (NC) group was examined under a microscope (Figure 4(a)), it was observed to have follicles present at different developmental stages, which were not observed with the PCOS group. Whether the PCOS group contained numerous cystic follicles (Figure 4(b)) is examined. The examination of the control group confirmed a normal ovarian tissue with the presence of developing follicle along with atretic follicle, primary follicle, and corpus luteum, whereas similar structures were observed with the plant extract tissue slide as observed in Figure 4(c). For a better outcome of the results, as described in the Materials and Methods, bitter melon extract was administered in combination with metformin in Figure 4(d). The stained tissue slides depicted some of the major stages of development of a follicle necessary for the normal reproductive cycle in females. The corpus luteum can be clearly seen, which is absent in the PCOS ovary. Moreover, the presence of atretic follicle, primary follicle, and developing follicle is also a confirmation of the ovary from the recovery of PCOS. On the other hand, the metformin group (Figure 4(e)) showed the presence of all the stages of a follicle under development mainly developing follicle, primary follicle, and also corpus luteum.

#### 3.2.3. Variation in Body Weight of Female Rats

During the initial PCOS induction phase, there was an increase in the body weight of both N.C and PCOS groups. But the PCOS group weight increase was double that of the N.C group. During the next four-week treatment phase, there was also variation in weight of the animals. PCOS group weight continuously increased significantly (*p* < 0.05) as compared to the control group, while the combination and metformin groups' body weight reduced significantly (*p* < 0.05) as compared to PCOS group. Body weight variation of animals is given in Figure 5.

#### 3.2.4. Effect of Aqueous Methanolic Extract of Bitter Melon (*Momordica charantia* L.) on Hormonal Levels

It was observed that, in the PCOS group, the testosterone level was significantly (*p* < 0.001) increased, while its level was decreased significantly (*p* < 0.001) in bitter melon, combination and metformin groups as compared to the PCOS group (Figure 6(a)). Similarly, the luteinizing hormone (LH) levels were significantly (*p* < 0.001) enhanced in PCOS group as compared to the normal group, but after treatment, a downfall in LH surge was found in all the treatment groups, and the most significant effects were observed in the combination and metformin group (Figure 6(b)), while the FSH level of the PCOS group was decreased significantly (*p* < 0.01) as compared to the control group. But after treatment, a significant (*p* < 0.001) improvement was observed only in the combination group of both bitter melon and metformin (Figure 6(c)). When the progesterone level was observed, a significant (*p* < 0.001) decrement was found as compared to normal control, but after treatment, we have found a significant incremental effect in all the treatment groups (Figure 6(d)). PCOS is a metabolic syndrome, and insulin resistance plays a major role in its pathogenesis. The PCOS group showed a significant (*p* < 0.001) increase in serum insulin levels. The combination group showed the most promising effects in reduction of insulin levels, and similarly, bitter melon and metformin also showed a significant reduction (Figure 6(e)).

#### 3.2.5. Effect of Aqueous Methanolic Extract of Bitter Melon (*Momordica charantia* L.) on Lipid Profile

PCOS perturbed the lipid profile, and most of the time, all the cholesterol parameters are changed with the progress of this morbid syndrome. In the present study, total cholesterol (TC) was increased significantly (*p* < 0.001), and similar type of effects was also in the case of triglyceride (TG) and low-density lipoproteins (LDL), while high density lipoprotein (HDL) level was reduced significantly (*p* < 0.001) as compared to the control group. However, all the treatment groups lowered down all of these, such as TC, TG, and LDL. HDL levels were improved significantly in the case of bitter melon, but this improvement was nonsignificant in the case of combination and metformin groups. Results are shown in Figure 7.

#### 3.2.6. Effect of Aqueous Methanolic Extract of Bitter Melon (*Momordica charantia* L.) on Antioxidant Enzymes

Superoxide dismutase (SOD) and catalase (CAT) are among the group of enzymes that have a role in cellular protection against the reactive oxygen species (ROS). Both are used as antioxidant markers. When SOD and CAT levels were determined by using liver homogenate, we found that both were decreased significantly (*p* < 0.001) after the induction of disease. But their level was significantly decreased after treatment with bitter and metformin and combination of both. Results are depicted in Figure 8.

#### 3.2.7. DPPH Assay

Antioxidant assay of the aqueous methanolic extract of bitter melon (*Momordica charantia* L.) was performed by using DPPH analysis method. Percentage inhibition of DPPH by bitter melon extract and butylated hydroxytoluene (BHT) was determined. Samples were taken in parts per million (PPM). BHT was used as a stand for comparing purposes. Results are shown in Table 3.

## 4. Discussion

PCOS is considered to be a complicated multigenic disorder that affects female population. Some of the most common features of PCOS include hirsutism, facial acne, and uncontrolled weight gain [39]. Hyperandrogenism is one of the major authentication factors for PCOS. PCOS has been a hallmark for an ovulary infertility in women [40]. The disorder has also been linked to irregular menstrual cycle in women of the reproductive age. Enlarged ovaries and presence of cysts are some of the most vital features of PCOS. This metabolic disorder is also linked with increased insulin resistance, which results in increased blood glucose levels [41].

Female reproductive organs, ovaries, are responsible all the events responsible for reproduction. The reproduction phenomenon is started with formation of ovum. The most initial phase is the follicles that mature into eggs. Hypothalamic gonadotropin-releasing hormone (GnRH) is responsible for regulation of pituitary hormones, for example, FSH and LH [42]. Unfortunately, in PCOS, this regulation is disturbed, and LH surge took place that depletes FSH and alters LH/FSH ratio. Due to this surge, more testosterone is produced, which leads to elevated level of Anti-Müllerian Hormone (AMH). Many follicles are present but have growth arrest and inability for enough maturation that leads to ovulation [43]. PCOS is heterogenous disorder that mostly happens in early-to-late reproductive age in females. There are multiple factors that have a role in pathogenesis of PCOS such as diet, lifestyle, genetic makeup, stress full life events, and many more.

Here, in the present project, standardized aqueous methanolic extract of bitter melon (*Momordica charantia* L.) was used for the management of PCOS. Extract is used alone and in combination with metformin. HPLC analysis revealed the presence of various phytoconstituents such as quercetin, gallic acid, benzoic acid, chlorogenic acid, syringic acid, *p*-coumaric acid, ferulic acid, and cinnamic acid; see Figures 1 and 2. PCOS was induced by using letrozole (1 mg/kg *p.o*.) for a period of four weeks. Letrozole, being an aromatase inhibitor, reduces the conversion of androgens to estrogens in the body [44]. Thus, in this way, it reduces the uterine weight and also reduces the LH surge and helps in induction of ovulation. But for disease induction, letrozole is used in low dose for 3–4 weeks; this is an effective model for disease induction and used by many researchers [45].

Actually, in PCOS, multiple follicles are present, but none will go into mature phase. An increase in weight was also observed during disease induction phase (Figure 5), and further confirmation of the disease is done by vaginal smear cytology. The presence of leucocytes and mucus showed the arrest of estrus cycle at diestrus phase; see Figure 3. Further confirmation was done by the histopathological analysis, multiple cystic follicles in ovaries of female rats, while the aqueous methanolic extract of bitter melon showed the follicles at various stages such as atretic follicle, corpus luteum, and developing and the primary follicle. The combination group also showed atretic follicle, corpus luteum, and developing and the primary follicle. The metformin group showed the presence of developing and primary follicle and corpus luteum; see Figure 4.

As discussed above, hypothalamic pituitary axis (HPO axis) plays an important role, and LH surge leads to FSH depletion, which has positive feedback on GnRH, which worsens the situation by releasing more LH, and this abnormality continues in PCOS [46]. It is the same phenomenon we observed on our PCOS female rats mode, elevated levels of LH and lower levels of FSH. When the treatment was deployed to PCOS rats, it reverts the situation by decreasing LH/FSH ratio and negative feedback on GnRH. Thus, FSH levels improved in all the treatment groups; see Figure 6. One another important factor is insulin resistance, which is evidenced with elevation of insulin levels in PCOS group. This is responsible for enhancing androgen levels [47]. We have also observed increased levels of testosterone in PCOS group, but treatment with bitter melon, combination, and metformin reduced these levels, which might be due to the overcoming insulin resistance and insulin surge down; see Figure 6.

The previous published data elaborated that quercetin can interact with LH and, in this way, inhibit androgen biosynthesis. Quercetin decreased LH and testosterone that is associated with regulation of steroidogenesis [48]. Additionally, gallic acid has also been previously reported to regulate the LH surge and rectify the irregularity of FSH in PCOS animals' studies [49]. Additionally, other phytochemicals such as *p*-coumaric acid and ferulic acid have a role in managing this disorder because of their ability to reduce the oxidation status and decremental effects on inflammation. [50, 51].

This study showed that bitter melon decreased serum levels of total cholesterol, TGs, and LDL, while it increased HDL levels (Figure 7). This change might be due to quercetin as well as other phytoconstituents present in the extract [48]. Kim and colleagues described the mechanism how quercetin reduced triglyceride level in obese patients [52]. Quercetin restricted the hepatic triglycerides accumulation by enhancing the hepatic mitochondrial oxidative metabolic capacity, which results in subsequent reduction of FFA induced lipid peroxidation. Moreover, it halts mitochondrial damage and hepatic lipid accumulation. Hyperglycemic is also one of the comorbidities of PCOS, and insulin resistance is the major cause. Evidence suggested that bitter melon may also have hypoglycemic effects [19].

Oxidative stress also has a role in pathogenesis of PCOS, and stress markers are. most of the time, elevated in PCOS females [9, 51]. Oxidative stress is actually the imbalance between the oxidants and antioxidants. PCOS is related to an oxidative state. Oxidative stress and various other conditions like IR, obesity, and abdominal adiposity and hyperandrogenism are comorbid [53, 54]. We also observed the elevated levels of SOD and CAT in PCOS rats. Many herbal remedies are there, which are effective in reducing the oxidative stress markers, for example, *Panax ginseng*, *Olea europaea, Bambusa arundinacea, Tinospora cordifolia,* and many other plants that have the antioxidant potential [55–57]. Similarly, bitter melon, combination, and metformin groups reduced these oxidation markers level depicting the positive impact on oxidation status (Figure 8). Moreover, bitter melon (*Momordica charantia* L.) extract has DPPH radical scavenging capacity 63.87% as compared to BHT (88.89%), which is used as a standard (Table 3). This is possible due to phenols and flavonoids rich extracts. Most of these phytochemicals present in extract have an excellent antioxidant potential [38, 54, 58].

The current study showed that treatment with bitter melon decreased insulin resistance. Thus, aqueous methanolic extract of bitter melon (*Momordica charantia* L.) has the potential to ameliorate PCOS. Furthermore, this study can be protracted to find out the effects of aqueous methanolic extract of bitter melon (*Momordica charantia* L.) at the molecular and genetic level.

## 5. Conclusion

The current study exhibited that aqueous methanolic extract of bitter melon (*Momordica charantia* L.) has the potential to ameliorate PCOS at the dose of 500 mg/kg, which was statistically comparable with metformin. Combination of bitter melon and metformin had synergized the beneficial effects. This property might be attributed to the direct effects of phytochemical like quercetin, gallic acid, benzoic acid, *p*-coumaric acid, and indirect effects as antioxidant and anti-inflammatory activities. Moreover, improvement in lipid profile, along with normalization of hormonal enzymes, might also play an important role in the overall management of PCOS and improve the symptomatology. Here, in this study, we provided the scientific data and proved that bitter melon has a potential to manage the PCOS. This study can be further elaborated at a molecular genetic level to strengthen the findings before the use for patient benefit.

## Figures and Tables

**Figure 1:** HPLC chromatogram of aqueous methanolic extract of bitter melon (*Momordica charantia L.*).

**Figure 2:** Structures of phytoconstituents present in aqueous methanolic extract of bitter melon (*Momordica charantia L.*).

**Figure 3:** The stages of estrous cycle in rats for 28 days in Normal Control and PCOS induced group.

**Figure 4:** Effect of aqueous methanolic extract of bitter melon (*Momordica charantia* L.) on ovarian tissues of PCOS induced female rats' model. Ovarian cross section stained by Hematoxylin-Eosin stain. (a) The control group showing the atretic follicle, corpus luteum, developing and primary follicle and oocyte (b) The PCOS group showing cystic and atretic follicles. (c) The bitter melon group can be observed with the follicles of various stages present such as atretic follicle, corpus luteum, developing and the primary follicle. (d) The combination group also showed atretic follicle, corpus luteum, developing follicles and the granulosa cells. (e) The metformin group is showed the presence of developing, atretic follicles, granulosa cells, primary follicle and corpus luteum. CL : Corpus luteum, Oo: oocyte, CF : Cystic follicles, AF: atretic follicles, DF: developing follicles, PF: primary follicles, GC: granulosa cells. Scale bar is equal to 100 *µ*M. Magnification 4×.

**Figure 5:** Effect of aqueous methanolic extract of bitter melon (*Momordica charantia* L.) on body weight (grams) in letrozole-induced PCOS female rats. Values are expressed as mean ± SEM (*n* = 5). Comparison among groups was done by using two-way ANOVA followed by Tukey's multiple comparisons test.  ^*∗*^*p* < 0.05;  ^*∗∗*^*p* < 0.01;  ^*∗#*^*p* < 0.05;  ^*∗∗#*^*p* < 0.01;  ^*∗∗∗###*^*p* < 0.001. ^*∗*^significant difference from Normal Control. ^#^significant difference from PCOS group.

**Figure 6:** Effect of aqueous methanolic extract of bitter melon (*Momordica charantia* L.) on various hormones. (a) Testosterone. (b) LH. (c) FSH. (d) Progesterone. (e) Insulin level, in letrozole-induced PCOS female rats. Values are expressed as mean ± SEM (*n* = 5). Comparison among groups was performed by using one-way ANOVA followed by Tukey's multiple comparisons test.  ^*∗#*^*p* < 0.05;  ^*∗∗#*^*p* < 0.01;  ^*∗∗∗###*^*p* < 0.001. ^*∗*^significant difference from Normal Control. ^#^significant difference from PCOS group.

**Figure 7:** Effect of aqueous methanolic extract of bitter melon (*Momordica charantia* L.) on lipid profile, in letrozole-induced PCOS female rats. Values are expressed as mean ± SEM (*n* = 5). Comparison among groups was performed by using two-way ANOVA followed by Tukey's multiple comparisons test.  ^*∗*^*p* < 0.05;  ^*∗∗*^*p* < 0.01;  ^*∗#*^*p* < 0.05;  ^*∗∗##*^*p* < 0.01; ^*#*^^*∗∗∗###*^*p* < 0.001. ^*∗*^significant difference from Normal Control. ^#^significant difference from PCOS group.

**Figure 8:** Effect of aqueous methanolic extract of bitter melon (*Momordica charantia* L.) on anti-oxidant enzymes. (a) SOD and (b) CAT, in letrozole-induced PCOS female rats. Values are expressed as mean ± SEM (*n* = 5). Comparison among groups was performed by using two-way ANOVA followed by Tukey's multiple comparisons test.  ^*∗*^*p* < 0.05;  ^*∗∗*^*p* < 0.01;  ^*∗#*^*p* < 0.05;  ^*∗∗##*^*p* < 0.01;  ^*∗∗∗###*^*p* < 0.001. ^*∗*^significant difference from Normal Control. ^#^significant difference from PCOS group.

**Table 1:** Experimental design and dosage schedule.

Groups	Treatment protocols
Normal control (NC) or control	Aqueous solution of carboxyl methylcellulose CMC 0.5% solution (10 mL/kg/day, *p.o.*)

Disease induced (PCOS)	Letrozole (1 mg/kg/day, *p.o.*) dissolved in CMC solution

Aqueous methanolic extract of bitter melon group *(Momordica charantia* L.)	Bitter melon extract (500 mg/kg/day, *p.o.*) dissolved in CMC solution

Bitter melon plus metformin) (combination group)	Bitter melon extract (500 mg/kg/day, *p.o.*) + metformin (500 mg/kg/day *p.o.*) dissolved in CMC solution

Metformin group	Metformin (20 mg/kg/day *p.o.*) dissolved in CMC solution

**Table 2:** HPLC analysis of phytochemicals present in aqueous methanolic extract of bitter melon (*Momordica charantia* L.).

Chemical constituents	Retention time (min)	Absorption rate PPM
Quercetin	2.880	76.53
Gallic acid	4.527	63.11
Benzoic acid	14.813	65.72
Chlorogenic acid	15.627	28.54
Syringic acid	16.307	11.06
*p*-coumaric acid	17.933	4.51
Ferulic acid	22.020	3.62

**Table 3:** DPPH scavenging potential of aqueous methanolic extract of bitter melon (*Momordica charantia* L.).

Aqueous methanolic extract of bitter melon (*Momordica charantia* L.)		BHT	
Sample PPM	Scavenging %	Sample PPM	Scavenging %
20	49.56	20	56.67
40	54.71	40	64.43
60	57.45	60	78.67
80	59.78	80	86.22
100	63.87	100	88.99

DPPH: 2,2-diphenylpicrylhydrazyl; BHT: butylated hydroxytoluene.

## Data Availability

The data used to support the findings of this study can be obtained from the corresponding author upon reasonable request.
